# River Pollution by Heavy Metals and Associated Impacts on the Adjacent Community, the Case of Holeta and Golli Rivers, Holeta Town, Ethiopia

**DOI:** 10.1155/2022/8064816

**Published:** 2022-08-30

**Authors:** Mathewos Temesgen, Abebe Shewamolto

**Affiliations:** Department of Biology, Ambo University, Ambo, Ethiopia

## Abstract

This study aimed to determine the level of heavy metals in the Holeta and Golli rivers and their impacts on the community of Holeta town, Ethiopia. Water samples were collected from eight randomly selected locations (4 sites from each river). A questionnaire survey, FGD, and KII were also used. Secondary data were also taken from the nearby health center. The flame atomic absorption spectrometer was used to analyze the samples. Fe, Mn, Ni, Cr, Pb, Cu, Zn, Co, and Cd were the identified heavy metals. The Holeta River contains Fe > Mn > Zn > Ni > Cr > Cu > Pb > Co > Cd, whereas the Golli River contains Fe > Mn > Zn > Ni > Cr > Cu > Pb > Co > Cd. The levels of Fe, Cr, Ni, Fe, and Mn were above the permissible limit of WHO (1984) and USEPA (1992). The primary sources of income for the people who lived in the area were farming and jobs on flower farms. Wastewaters discharged from the surrounding flower farms were the major polluting source (84.3%) of the river. About 84.3% of the surrounding community claimed that wastewaters discharged from the flower farms are the major polluting sources of both rivers. Many of the flower farmworkers (43.9%) have also exposure to toxic insecticides and pesticides used on the farm. About 60% and 20.5% of the workers have frequent severe headaches and skin irritation due to exposure to heavy metals. Generally, both the surrounding community and flower farmworkers are facing significant health and socioeconomic impacts due to the heavy metals joining the rivers. Therefore, effective management of pollution sources and continuous monitoring of the river quality is very imperative to minimize the impacts.

## 1. Introduction

Heavy metals are a major class of pollutants in our world arising principally from natural and anthropogenic sources [1]. They are a group of metals and metalloids with relatively high atomic mass (>4.5 g/cm^3^) and are toxic even at low concentrations [2]. The chief heavy metals noted in the environment include mercury (Hg), cadmium (Cd), arsenic (As), chromium (Cr), thallium (TI), lead (Pb), copper (Cu), manganese (Mn), zinc (Zn), and nickel (Ni). Most of them are essential micronutrients for plants, animals, and humans, but at high concentrations, they may cause toxicity and harm animals' health including human beings because of their nonbiodegradable nature, which causes them to readily accumulate in tissues and living organisms [3]. Of these, Hg, Pb, Cd, and As are recognized as health hazards, and all of them cause major health problems [4]. They accumulate in the food webs mainly in fishes and vegetables and then threaten the living organisms that depend on these groups for their foods [5].

The exposure of humans to heavy metals can occur through a variety of routes, which include inhalation as dust or fumes, vaporization, and ingestion through foods and drinks [6]. Workers who have exposure to different chemicals used in industry and enclosed spaces can also be exposed to heavy metals through the skin and inhalation [7]. Besides, toxic chemicals such as pesticides and fertilizers can migrate via water into the food chain and be consumed by humans and animals through foods [8].

Most of the industries in the developing countries are discharging their wastes directly into the nearby streams, rivers, lakes, oceans, and open lands without any treatment [9]. Moreover, heavy metals are not subjected to bacterial degradation and hence remain permanently in the aquatic environment [10]. Contamination of rivers with these metals may cause devastating effects on the ecological balance of the aquatic environment and the diversity of aquatic organisms [11]. The chronic level ingestion of toxic metals has also undesirable impacts on humans, and the associated harmful impacts are visible after several years of exposure [3, 12]. Therefore, a better understanding of heavy metal sources, their accumulation levels in the rivers, and their effects on human health seem to be important issues in present-day research work [13].

Holeta Town is one of the industrial zones located in the western part of Addis Ababa, Ethiopia. It is characterized by the rapid expansion of floriculture industries in recent years with extensive use of the river's water, fertilizers, and pesticides in flower farms [14]. The effluents from the flower farms are discharged into a channel that flows through the nearby rivers including the Holeta and Golli rivers. However, there is no scientific information on the level of heavy metal pollutants in the adjacent rivers and the impacts of these metals on the society living near the river. This study was therefore aimed to analyze the level of the heavy metal pollutants in the Holeta and Golli rivers, and their impacts on the community living in the area.

## 2. Materials and Methods

### 2.1. Description of the Study Area

The study was conducted at Holeta and Golli rivers around Holeta Town, Walmara District, Ethiopia (Figure 1). The town is located in the Special Zone of Oromia National Region State Surrounding Finfine (SZOSF) at a distance of 29 km from the capital Finfine toward the west direction on the main road to Ambo-Nekemte. The town is located at a latitude of 9°01′08″ to 9°06′15″N and longitude of 38°26′40″ to 38°32′46″E (Annual plan of Holeta town, 2019). The town covers about 61.5 km^2^. Topographically, it is characterized by dissected plateaus, plains, and valleys. The agro-climatic zone of the town is the middle land (Woyna Dega) with minimum and maximum temperatures of 21°C and 1.7°C, respectively. The annual rainfall also ranges between 900 and 1100 mm with a bimodal rainfall pattern. The town receives the highest rainfall in the months from July to August. The area is characterized by major land use and land cover types such as agricultural land, forest, pasturelands, settlement areas, water bodies, and barren lands. Holeta River is the river that crosses the town and flows with the south direction in Sadamo Kebeles, whereas the Golli River flows in the west direction from the Holeta town at the periphery of Galgal Kuyu kebele.

### 2.2. Research Design and Data Sources

A mixed research design approach that involves both qualitative and quantitative data collection methods was performed. Both primary and secondary data collected from different sources were used. Primary data were gathered from the water samples collected from Holeta and Golli rivers. The information regarding the impact of heavy metals on the community was collected from the residents living near the river and from the employers of the floriculture industry enterprises. The secondary data were also collected from nearby health centers.

### 2.3. Sample Site Selection

Holeta and Golli Rivers were purposely selected for this study because these rivers are extremely deteriorated by effluent that discharges from the nearby flower farms. A preliminary survey was made in the study area from January through February 2012 to get important information regarding the study area, which helped to select the sampling sites. Eight sampling sites were selected randomly from the two rivers for water sample collection four sites from each river following the longitudinal gradient of the rivers based on the information obtained in the preliminary survey (Table 1).

In addition, three peasant associations (locally called kebeles), namely, Burka Walmara, Sadamo, and Galgal Kuyu, were selected purposely for the questionnaire surveyed from the eight kebeles of the town because the three kebeles have direct contact with the two rivers and wastewater discharging from the flower farms.

### 2.4. Sample Size Determination for Questionnaire Survey

A total of 3248 household heads were living in the three kebeles (Table 2). In addition, 600 employers were working in the three selected flower farms during the data collection (Table 3). The sample size of the respondents to be involved in the questionnaire survey was estimated using the [15] formula, which was calculated as follows:

(1) $$\begin{array}{c} n=\frac{N}{1}+N^{2}{}_{e}, \end{array}$$

where *n*  denotes sample size, *N*  denotes total population, and *e*  denotes precision level.

Using 0.07 percent of the margin of error, the total sample size of the respondents was as follows:

(2) $$\begin{array}{c} n=\frac{3248}{1}+3248{\left(0.07\right)}^{2}. \end{array}$$

Thus, a total of 159 respondents were randomly selected from the three kebeles. A proportionate sampling method was used to select the household respondents in each kebele using *n*^*∗*^*N*/*T*, where *n* is the total sample size from the three kebeles, N is the total number of household heads in each kebele, and *T* represents the total number of household heads in the three kebeles (Table 4).

In addition, the flower farm employers were engaged in the questionnaire survey. The sample size of the respondents from the flower farmers was also calculated using the [15] formula as *n* = 600/1 + 600(0.07)^2^ using a 0.075 percent of margin of error. The total number of respondents involved from the employers was 132. The number of respondents from each farm was also calculated using *n*^*∗*^N/T, where *n* is the total sample size from the three flower farms, N is the total number of workers in each flower farm, and *T* represents the total number of workers in the three flower farms (Table 3).

### 2.5. Data Collection Techniques

#### 2.5.1. Water Sample Collection

Before sample collection, the bottles were thoroughly washed with detergent, rinsed with distilled water, and soaked in 2% HNO_3_ for each sample. A composite of 1000 ml of water samples was collected from each site using polyethylene plastic bottles with a replicate. The samples were kept in green plastic bottles and transported to Holeta Agricultural Research Institute for laboratory analysis. The samples were stored at room temperature (refrigerator 4°C) before laboratory analysis.

#### 2.5.2. Data Collection for the Impacts of Heavy Metal Pollutants

Open- and close-ended questionnaires were used for data collection on the impact of heavy metal pollution on society. The questionnaires were prepared in English and translated to Afaan Oromo, for further communication with the respondents. The questionnaires were pretested among some groups, which were not included in the primary study for validation of the contents. Then, the questionnaires were distributed to the respondents after modification was made based on the feedback obtained from the pretested questionnaires.

### 2.6. Laboratory Analysis

#### 2.6.1. Water Sample Preparation

For digestion of the samples, 50 ml of each water sample was taken and 5 ml of HNO_3_ was added to remove microorganisms. A 25 ml of the samples was then taken after being freed from microbes and heated at 80°C to split the compound into elements.

#### 2.6.2. Instrumental Calibration

Intermediate standard solutions (100 mg/L) of each metal were prepared from stock standard solutions containing 1000 mg/*L* of Cd, Cr, Pb, Cu, Zn, Fe, Cr, Co, and Mn. Appropriate working standards were prepared for each of these metal solutions using a dilution of the intermediate solutions using distilled water in 2N HNO_3_. Using the instrument operation manual, to attain its better sensitivity, the working standards were aspirated one after the other into the flame atomic absorption spectrometry (FAAS) and their absorbance was recorded. Calibration curves were plotted with different points for each of these metal standards using absorbance against concentration (mg/L). Immediately after calibration, the sample solutions were aspirated into the FAAS instrument and a direct reading of the metal concentrations was made (Table 4).

#### 2.6.3. Continuing Calibration Standards (CCS)

Continuing calibration standards (CCS) were used to verify the calibration accuracy during every analytical run. The CCS was prepared from the midpoint of the initial calibration standard of metal analysis. CCS was verified after every nine measurements for each analysis.

#### 2.6.4. Analysis of Heavy Metals

First, the instrument was calibrated with a calibration blank and nine series of calibration standard solutions. The instrument was then fitted with a specific lamp of a particular metal. Air-acetylene, fuel-oxidant mixture, was used as the fuel and the air as it passed in the standard method. The levels of heavy metals were identified using AAS (Agilent Technologies, 200 Series AA) following the APHA (1999) standard method.

### 2.7. Data Analysis

The data collected were fitted into MS Excel and edited before statistical data analysis. Student's t test was used for statistical testing of the heavy metal concentration difference among the study rivers at *p* < 0.05 and *p* < 0.01 significant levels using SPSS 22 software. All results were reported as mean ± standard deviation of double measurements. Descriptive statistics were also performed to analyze the results obtained from the questionnaire survey, and the results were presented in figure and table form.

## 3. Results

### 3.1. Level of Heavy Metals in Water Samples

A total of nine heavy metals (Fe, Mn, Ni, Cr, Pb, Cu, Zn, Co, and Cd) were identified from the total water samples. The content of Pb, Ni, Mn, Fe, Co, and Cr was higher in the water samples collected from the Holeta River, whereas Cu, Zn, and Cd were higher in the Golli River. The level of heavy metals indicated that Fe > Mn > Zn > Ni > Cr > Cu > Pb > Co > Cd in the water samples collected from Holeta River, whereas Fe > Mn > Cu > Zn > Cr > Ni > Co > Pb > Cd in the Golli River (Table 5). Except for Ni and Fe (*p* < 0.05), the level of heavy metals did not show a significant difference (*p* > 0.05) between the two rivers, but a significant spatial variation was observed in each of the study rivers (*p* < 0.05).

Except for Cd and Fe, the results also revealed that all detected heavy metals in both rivers had positive relationships with one another and the correlations were statistically significant for most of the heavy metals (Table 6).

### 3.2. Assessment on the Impacts of Heavy Metals

#### 3.2.1. Socio-Demographic Characteristics of the Respondents

A total of 291 respondents were involved in this study. Of these, 48.1% were males and 51.9% were females. One hundred and thirty-two respondents (63.6% females and 36.4% males) were flower farm workers and 159 (57.7% males and 40.3% females) were from the community living near the rivers. The majority of the respondents from the two categories fall in the age range of 20–30 years old with a mean age of 27.6 years. The majority of the flower farm workers involved in the study were illiterate (22.7%), whereas 94.97% of the community was able to read and write. About 60.6% of the flower farm workers and 59.7% of the surrounding community were married, but 44.7% and 42.78% of them had no children. About 40.2% of the flower farm employers came from other areas; and all of them were completely dependent on the flower farm for their livelihood, whereas 94.7% of them were permanent workers. In other ways, 42.76% of the local community was completely dependent on agriculture (Table 7).

#### 3.2.2. The Impact of Heavy Metal Pollutants on the Flower Farm Workers

About 43.9% of the workers had direct exposure to all chemicals used in the flower farms, and 77.3% of them did not wear any safety materials during their work time. Severe frequent headaches (35.6%) and skin rash or irritations (26.5%) were the major problems facing the workers since they started to work on the farm. For about 70.5% of the employers, the chemicals used on the farms were the reason for their health-related problems (Table 8).

About 28.8% of the workers spend more than 500 ETB (12.5 USD) per month for medical treatment at the Holeta Health Center or other medical centers due to the problems associated with the flower farm chemicals (Figure 2).

About 84.8% of the workers did not have a regular medical checkup at the farm, but they always have exposure to chemicals like fungicides, insecticides, and fertilizers while they worked on the farms. About 62.1% of the farmers did not also get any kind of assistance during their entire work time from the companies for their health-related problems (Figure 3).

The management practices of heavy metals/pollutants impacting on the workers were only shifting the workers from one work position to the other (23.48%) or giving rest for the workers when they are sick (21.94%) (Figure 4).

#### 3.2.3. The Impact of Heavy Metal Pollutants on the Surrounding Society

About 47.8% of the community uses the river's water for irrigation after the wastewater discharged from the flower farms joins the river, whereas 40.9% of them use it for drinking. About 78.0% of the community confirmed a significant recent color change on the river due to the effluents joining the river from the flower farms (Figure 5).

Death of livestock dermatitis and decreasing agricultural production due to not being interested in using the river water for irrigation were the major problems for about 74.2% of farmers living in the study area (Figure 6).

#### 3.2.4. Diseases Frequently Affect Livestock

Dermatitis/skin disease was the major problem affecting the livestock (51.3%) in the vicinity of the rivers followed by internal diseases (34.2%) (Figure 7).

The mean per capita loss due to the expenses for treating their livestock was estimated to be 757.6 ± 253 ETB (18.7 USD). In this regard, the total annual loss for all respondents due to the expenses of treating their livestock was 47728.8 ETB (1178.5 USD). In addition, the mean per capita loss due to death of livestock was estimated to be 20,000 ± 4000 ETB (493.8 USD) and the total estimated annual loss for all respondents was about 220,000 ETB (5432.1 USD). The overall estimated loss due to treating livestock and the death of livestock within five years was 267,728.80 ETB (6610.6USD) (Table 9).

## 4. Discussion

### 4.1. Heavy Metal Concentration in the River Water

Heavy metal contamination is a major problem for the environment, especially for rapidly growing cities in developing countries due to uncontrolled pollution levels driven by many causative factors [6]. Flower farms use various chemicals in the form of fertilizers and pesticides, which can be easily washed off and enter the water bodies [8]. Holeta and Golli rivers are the rivers that are located at point sources of pollution in the periphery of flower farms in Holeta town. The rivers are highly polluted due to the discharging of wastewaters from flower farms such as Oromia Wanders PLC, Ethio-dream PLC, and Euro-flora PLC, which accounted for heavy metal pollution in both rivers.

In this study, a total of nine heavy metals were identified. The levels of heavy metal content were higher in the Holeta River than in the Golli River. This could be attributed to the high density of flower farms around the Holeta River. This is in agreement with the findings of [16], who reported the high density of flower farms in the Upper Awash Valley, around Lake Ziway, Sebeta town, Bishoftu town, and Addis Alem town with a prominent pollution impact on the nearby rivers.

Iron is the most abundant and essential element for all plants and animals. Perhaps, it may cause tissue damage and some other diseases in humans at high concentrations [17]. The mean concentrations of Fe in both rivers were higher than the recommended limit of [18] (0.3 mg/l) in the drinking water. It is also higher than the finding of [19] from the Rebu River (2.02 mg/l). The high content of Fe in both rivers indicates the pronounced impact of flower farms on the rivers [8, 20].

Manganese is also an essential element required for various biochemical processes like normal bone structure, reproduction, and normal functioning of the central nervous system [21]. Overconsumption of Mn, however, causes both mental and emotional disturbances along with an increased slowness and clumsiness of body movements [22]. The mean contents of Mn recorded in both rivers were higher than the permissible limits of WHO [23] (3.3 mg/l) and WHO [18] (0.1 mg/l) in drinking water. It was also higher than the finding of Bedassa et al. [24] from the Mojo River (2.90 mg/l), Meki River (0.545 mg/l), and Ziway Lake (0.089 mg/l). It was however lower than the report of G/Wold et al. [25] (0.094 to 0.123 mg/l) from the Ogona River, Goba Town. The difference might be attributed to the variation in the level of pollution potential among the study areas, which may depend on the type of industry and the treatment method performed in the areas [26].

The mean concentrations of Ni recorded in both rivers were also higher than the permissive limit of USEPA [27] in drinking water (0.1 mg/l). It was however lower than the finding of Yohannes and Elias [26] in Bulbula River (74.13 mg/l).

Cr (III) and its compounds are not considered a health hazard, but the toxicity and carcinogenic properties of Cr (VI) have been well reported [28]. This is because Cr (VI) forms negatively charged species (HCrO_4_- or CrO4_2_-), which are relatively mobile. It has several health impacts such as ulcers, corrosive reactions on the nasal septum, acute irritative dermatitis, and allergic eczematous dermatitis [29]. Numerous studies have also shown that inhalation of Cr (VI) can cause lung cancer in humans [30]. The concentrations of Cr in both rivers of the present study were above the permissible level of Cr for drinking water (0.05 mg/l) [27]. This indicates that Cr is a potential health risk in the study area due to the presence of Cr in the water above the permissible limit [31]. It was also higher than the report of Wold et al. [32] (0.04 to 0.07 mg/l) from Ogona River of Goba Town, but lower than the report of Bedassa et al. [24] (2.039 mg/l) from Mojo River, where the lather industries are discharging the wastewater into the river.

Lead toxicity is also known to cause musculoskeletal, renal, ocular, neurological, immunological, reproductive, and developmental effects [33]. The Pb contents measured in the Holeta River were above the maximum permissible limit of Pb for drinking water (0.05 mg/l) [27]. It was however lower than the finding of Yohannes and Elias [26] from Bulbula River (14.10 kg/l) and Tadesse et al. [34] from Rebu River (0.16 mg/l).

Cadmium is also a highly toxic nonessential heavy metal, and it does not have any role in biological processes. Even at low concentrations, cadmium could be harmful to organisms [33]. Cd pollution causes anemia, renal damage, bone disorder, and lung cancer [35]. The mean concentrations of Cd in the Golli River were above the permissible limit for drinking water (0.005 mg/l) [36]. It was also higher than the finding of Yohannes and Elias [26] from the Bulbula River (0.07 mg/l).

### 4.2. The Impact of Heavy Metals on Flower Farm Workers

The means of livelihood of all workers were highly dependent on the income obtained from the flower farms. The workers also had high exposure to chemicals used on the farms, mainly insecticides and fungicides without wearing safety materials. Thus, they are frequently facing different health problems like severe headaches and skin rash or irritation. Most of the dermal effects and headaches observed might be associated with exposure to high levels of chromium compounds or other related heavy metals used in the farms [37,38]. The study also indicated that the provision of necessary facilities for workers such as showers, safety materials, washing facilities, and free medical services are inadequate, and the workers are highly affected with the chemicals used in the flower farms in Ethiopia [8,39]. In line with this finding, Dessalegn [40] also reported that about 90.6% of the workers had at least one sign and symptom of work-related health issues since they were employed on flower farms in the East Shewa Zone of Ethiopia. Abul [41] also revealed that asthma, branchiate infection, and skin irritation are the most frequently occurring diseases in the Ethiopian flower farm industry due to the high usage of heavy metals such as Cr, Mn, and Fe in the flower farms.

Due to the heavy metal impacts, the flower farmworkers are spending more than 500 ETB per month for their medical treatment. The study conducted in Uganda also revealed that the payment for the flower farmworkers is too small in comparison with the safety of workers and the economic situation in Uganda [42]. There was also no regular medical checkup and medical support offered to the workers. The study made in other parts of the Oromia Region also confirmed similar concerns in flower farms [39].

### 4.3. The Impact of Heavy Metal on the Surrounding Community

The community living near the two rivers was dependent on the rivers for irrigation, home consumption, and catering to their livestock. The flower farms present in the study area also release toxic chemicals into the rivers without any treatment. Moreover, children were more prone to this pollution since they were frequently playing around the rivers, and they had direct contact with the river, while they washed their clothes, swam, and drank the water. These were highly affecting the health of the community living in the area and their livestock. The studies also indicated that people living around flower farms and polluted rivers are very susceptible to river pollutants in different ways [7, 8, 25, 43].

The majority of the residents were complaining about the presence of flower farms around their area because they are releasing the waste into the rivers, farmlands, and grasslands without any treatment. This might be due to the lack of effective management setup and follow-up by all concerned bodies. The floriculture farms have the EIA on their hands, but they were not fully implementing the activities designed in their plan. The study also reported similar challenges in different parts of Ethiopia [8]. Our findings also revealed that farmers lost more than 16 major livestock within five years due to acute death associated with rivers' pollution, and spent a lot in treating their livestock due to different associated diseases, which is estimated to be about 267728.8 ETB in five years. UNESCO [44] also reported that due to water pollution and lack of sanitation, the overall economic loss is estimated to be 5% of the gross domestic product in Africa.

## 5. Conclusion

In this study, water samples analyzed for the assessment of heavy metal concentration showed the presence of toxic heavy metal pollutants (Cd, Ni, Cr, Fe, Pb, and Mn) in both rivers. The levels of these metals were beyond the maximum limit for drinking water and irrigation water. This is because some flower farms are discharging wastewater to the river without any treatment. Employers in flower farms are also highly exposed to the heavy metal pollutants used in the flower farms. The surrounding community was also facing serious health and socioeconomic problems due to direct and frequent exposure to river pollution. This calls for effective management of the pollutants at the pollution sources level and strengthens the integral work among all concerned bodies. [45]

## Figures and Tables

**Figure 1:** Map of the study area (source: Authors lab work, 2022).

**Figure 2:** The monthly expense of workers for medical treatment in the study area.

**Figure 3:** Opinion on the regular medical checkup and medical supports for the workers.

**Figure 4:** The management practices of heavy metals/pollutants impacts in the study area.

**Figure 5:** The contribution of the Holeta and Golli river waters for the surrounding community.

**Figure 6:** The impacts of rivers pollution on the adjacent community.

**Figure 7:** Diseases affecting the livestock in the study area.

**Table 1:** The selected sampling sites from the two rivers and their designation.

S N.	Name of the site	Coordinates	Characteristics
1	HR1	9°03'58.75 N and 38°30'56.38” E	The outlet at which the wastewater discharging from the Oromia wanders flower farm flows to Holeta River
2	HR2	9°03'58.23” N and 38°30'45.06”E	In the channel in which the wastewater flows from the Oromia wanders the flower farm drain before being mixed with Holeta River water 100 m from HR1.
3	HR3	9°04'09.03” N and 38°30'36.03”E	The site selected from Holeta River after effluent from the Oromia wanders flower farm joined the river 200 m from the joining site.
4	HR4	9°03'53.79”N and 38°30'39.05” E	The site was selected from Holeta River before the effluent from the Oromia wanders flower farm joined the river.
5	GR1	9°03'17.81”N and 38°27'20.07” E	The outlet at which the wastewater discharged from Euro flora flower farms flows to the Golli River.
6	GR2	9°03'18.93”N and 38°27'18.32 E	In the channel that drains the wastewater discharging from Ethio-dream and Euro flora flower farms before mixed with the Golli River on 200 m from GR1
7	GR3	9°03'39.46N and 38°27'21.59” E	The site was selected from the Golli River after the effluents from Ethio-dream and Euro flora flower farms mixed with the river 500 m from the joining site.
8	GR4	9°03'08.85”N and 38°27'19.73”E	The site was selected from Golli River before the wastewater discharged from the flower farms joined the river

**Table 2:** The total population and sample size of the respondents from the three study kebeles.

Kebeles	Total population of the kebele	Estimation of sample size	Sample size
Sadamo	1229	1229 × 159/3248 = 60	60
Galgal Kuyu	1523	1523 × 159/3248 = 75	75
Burka Walmara	496	496 × 159/3248 = 24	24
Total	3248		159

**Table 3:** Total population and sample size of the respondents from the three flower farms.

S.No	Name of flower farm	Total no. of flower farm workers	Estimation of sample size	Sample size
1	Oromia wonders PLC	360	132 × 360/600 = 78.6	79
2	Ethio-Dream flowers PLC	90	132 × 90/600 = 19.65	20
3	Euro flora PLC	150	150 × 131/600 = 32.75	33
Total		600		132

**Table 4:** Calibration graph absorbance against the concentration of heavy metals in mg/L.

S.No.	Metal	Model for Absorbance vs. concentration	R^2^
1	Zn	y = 0.3328*x*	0.9960
2	Cu	y = 0.0804*x*	0.9972
3	Mn	y = 0.0883*x*	0.9983
4	Cd	y = 0.1291*x*	0.9953
5	Cr	y = 0.0402*x*	0.9981
6	Pb	y = 0.0059x	0.9972
7	Ni	y = 0.0273*x*	0.9965
8	Co	y = 0.0198*x*	0.9976
9	Fe	y = 0.0163*x*	0.9986

**Table 5:** The level of heavy metal contents in water samples collected from Holeta and Golli rivers.

Metals (Mg/ L)	Holeta River (Mean ± SD)	Golli River (Mean ± SD)
Pb	0.05 ± 0.019a	0.02 ± 0.02a
Ni	0.19 ± 0 0.15a	0.16 ± 0.12b
Mn	3.8535 ± 3.31a	2.748 ± 2.63a
Fe	204.3200 ± 129.73a	60.1525 ± 37.68b
Co	0.0445 ± 0 0.04a	0.03 ± 0.02a
Cu	0.1053 ± 0.068a	2.4175 ± 0 2.36 a
Zn	0.6050 ± 0.29a	0.9725 ± 0.89 a
Cd	0.003 ± 0.003a	0.01 ± 0.0021 a
Cr	0.1805 ± 0.13a	0.1670 ± 0.15a

NB: the mean values of the same latter were not significantly different (*p* ≤ 0.05).

**Table 6:** The Pearson correlation test for the mean of each heavy metal in the water samples.

Metal	Pb	Ni	Mn	Fe	Co	Cu	Zn	Cd	Cr
Pb	1								
Ni	0.8788^*∗∗*^	1							
Mn	0.8080^*∗*^	0.9552^*∗∗*^	1						
Fe	0.584	0.682	0.7018^*∗*^	1					
Co	0.5325	0.7683^*∗*^	0.8378^*∗∗*^	0.4771	1				
Cu	0.7522^*∗*^	0.4647	0.5184	0.2253	0.2843	1			
Zn	0.7949^*∗*^	0.7052^*∗*^	0.7702^*∗*^	0.517	0.4808	0.8658^*∗∗*^	1		
Cd	0.2976	0.1707	0.1854	-0.4253	0.2625	0.607	0.478	1	
Cr	0.7464^*∗*^	0.8990^*∗∗*^	0.9438^*∗∗*^	0.6471	0.6868^*∗*^	0.5133	0.8326 ^*∗*^	0.2462	1

^*∗*^ indicates a significant correlation at *p*=0.05, and ^*∗∗*^ indicates a significant correlation at *p*=0.01.

**Table 7:** Socio-demographic characteristics of the respondents engaged in this study.

Socio-demographic characteristic	Category	Flower farms employers		The surrounding community		Total	
		*N*	Percentage (%)	*N*	Percentage (%)	*N*	Percentage (%)
Sex	Female	84	63.6	67	42.1	151	51.9
	Male	48	36.4	92	57.9	140	48.1
Age group	<20	2	1.5	4	2.5	6	2.1
	20-30	85	64.4	85	53.5	170	58.4
	31–40	29	22.0	31	19.4	60	20.6
	41–50	10	7.6	18	11.3	28	9.6
	>50	6	4.5	21	13.2	27	9.3
Educational level	Illiterate	30	22.7	8	5.0	38	13.1
	Adult education	22	16.7	11	6.9	33	11.3
	Primary school	28	21.2	18	11.3	46	15.8
	Junior school	18	13.6	22	13.8	40	13.7
	Secondary school	17	12.9	38	23.9	55	18.9
	Preparatory school	6	4.5	19	11.9	25	8.6
	Diploma	9	6.8	31	19.5	40	13.7
	Degree and above	2	1.5	12	7.5	14	4.8
Marital status	Single	41	31.1	62	39.0	103	35.4
	Married	80	60.6	95	59.7	175	60.2
	Divorced	8	6.1	0	0.0	8	2.7
	Widowed	3	2.3	2	1.3	5	1.7
Number of children	No children	59	44.7	68	42.8	127	43.6
	1-3	46	34.8	48	30.2	94	32.0
	4-6	8	6.1	2	1.3	10	3.4
	> 6	19	14.4	41	25.8	60	20.6
Occupation	Private	132	100.0	134	84.3	266	91.4
	Farmer	0	0.0	68	42.8	68	23.4
	Trade	0	0.0	30	18.9	30	10.3
	Governmental	0	0.0	25	15.7	25	8.6
Mean of livelihood	Private works	132	100.0	38	23.9	170	58.4
	Governmental workers	0	0.0	23	14.5	23	7.9
Type of employment	Permanent	125	94.7	0	0.0	125	94.7
	Part time	1	0.8	0	0.0	1	0.8
	Occasional	6	4.5	0	0.0	6	4.5
Service years	1 year	21	15.9	0	0.0	21	15.9
	2 years	26	19.69	0	0.0	26	19.7
	3 years	27	20.45	0	0.0	27	20.5
	> 4 years	58	43.9	0	0	58	43.9

**Table 8:** The types of chemicals frequently exposed, means of keeping their safety and health problems of the flower farm workers.

Parameter	Category	Frequency	Percentage (%)
The type of chemicals workers frequently exposed	All kinds of chemical	58	43.9
	Insecticides and Fungicide	47	35.6
	Not interested to respond	20	15.2
	Fertilizers	3	2.3
	Insecticides	2	1.5
	Fungicides	2	1.5
Ways of keeping their work safety	Not wear safety materials	102	77.3
	Wear safety materials	30	22.7
The workers keeping their work safety	Frequent headache	47	35.6
	Skin rash or irritation	35	26.5
	Rapid weight loss	16	12.1
	Kidney problem	12	9.1
	Gynecological problem	10	7.6
	Asthmatics	8	6.1
	Persistent cough	4	3
The workers frequent health problem	Chemicals used in the farm	93	70.5
	Not interested to respond	28	21.2
	The work is tiresome	6	4.5
	Prolong working hours	4	3.0
	Lack of rest time	1	0.8

**Table 9:** The estimated loss of farmers due to treating and death of their livestock in the last five years (2016-2020).

Type of loss	Quantity	Money spent (ETB)	Mean ± SD	Total estimated loss (ETB)
		Range		
Treated livestock	63	500–1000	757.6 ± 253	47728.8
Death (livestock)	16	15000–23000	20,000 ± 4000	220000

## Data Availability

All the data used are presented in this article.
